# Semantic Analysis Technology of English Translation Based on Deep Neural Network

**DOI:** 10.1155/2022/1176943

**Published:** 2022-07-11

**Authors:** Qi Wang

**Affiliations:** School of Foreign Languages, Henan University of Animal Husbandry and Economy, Zhengzhou, Henan 450046, China

## Abstract

English translation plays an important role in the development of science and technology and cultural exchanges. With the increase in translation volume, intelligent translation has become inevitable, but there is no effective solution for semantic translation in English translation. To provide an effective translation improvement scheme in English translation, this paper studies and analyzes the application of deep neural network in English translation semantic analysis. Based on a brief analysis of the research progress of English translation analysis and the current situation of neural network, a neural network translation architecture is established, and a deep neural network model for English translation analysis is proposed. Aiming at the problem of gradient disappearance in RNN model, the ability of Gru neural network to deal with long-distance translation is enhanced, and the computational complexity of Gru neural network is reduced. At the same time, a bi-directional Gru model is designed to translate according to the context. For some nonlinear translation, a deep neural network model based on part of speech sequence information is proposed to realize semantic analysis, and experiments are designed to test the translation effect of the neural network model. The simulation results show that the English translation based on deep neural network can improve the translation effect, reduce errors and improve the accuracy of semantic analysis of English translation, which has certain reference significance for improving the level of English translation.

## 1. Introduction

In the field of artificial intelligence, English translation and even natural language processing are important courses. Language analysis can be realized through the communication between human and machine [1]. At present, the commonly used natural language translation is evaluated according to the neural network framework. Language translation is a cross science involving a wide range of fields. In addition to linguistics, it also involves the fields of mathematics, computer, and automation technology [2]. After years of development, the theory has gradually matured. In this application field, machine translation is an important part. At present, the common machine translation uses the neural network model to transform the language to be translated into another natural language. Its formation is based on mathematical computer technology [3]. Machine translation has developed in an all-around way in recent years. In addition to scientific research, people's livelihood has also begun to use this kind of translator [4]. However, the translation model based on neural network is not omnipotent. The performance of translation remains to be discussed, and the need itself is constantly changing. Therefore, the study of semantic analysis of English translation based on deep neural network has important practical significance for improving translation performance [5].

Based on this background, this paper studies the application of English translation semantic analysis based on deep neural network, which is mainly divided into four chapters. The first chapter briefly introduces the application research and current situation of natural language translator and briefly introduces the chapter arrangement of this paper; Chapter 2 introduces the application of machine translation and neural network research, and summarizes the shortcomings of the current research. In Chapter 3, based on the existing neural network model, the framework of encoder and decoder is constructed. Aiming at the shortcomings of cyclic network and long-term and short-term memory in the existing mainstream neural network translation, an independent cyclic neural network is proposed, and the part of speech sequence information is introduced, which is spliced with word vector and position vector as the common input information. In Chapter 4, the neural network translation model is simulated and analyzed to measure the translation performance and convergence. The experimental results show that the depth neural network proposed in this paper has better performance in resisting noise data, can improve the translation performance, reduce the translation error, and reduce the running time. The bidirectional Gru neural network model has certain advantages in English translation. In the convergence analysis, the loss function under rnnlm model decreases relatively slowly. After adding part of speech sequence information, the convergence speed of the loss function decreases faster, but the convergence effect is better than the traditional algorithm. In the translation of long sentences, the performance of several deep neural network translation models can improve the translation effect, but the superiority of the translation performance of the model with part of speech sequence information is more obvious.

The innovation of this paper lies in the application of part of speech sequence information. In view of the limitations of machine translation itself, combined with linguistic knowledge, and based on the previous research progress of neural network, a two-way Gru machine translation model is established to realize semantic translation and improve translation performance. At the same time, the part of speech sequence information is introduced into the two-way cyclic neural network model, and the background vector is spliced by two-way coding to improve the translation performance of the deep neural network model.

## 2. State of the Art

English is one of the international common languages. English semantic analysis plays an important role in the use, input, and translation of English. At the same time, it is also one of the basic technologies affecting English reading. In the current various translation models, semantic analysis does not consider the context and is vulnerable to noise interference. Many people have studied translation recognition. For example, Anderson et al. believe that compared with other learning algorithms, the use of neural network can reveal the distributed characteristics of sentence-level meaning of coded propositions [6]. Wang et al. pointed out in their research that most of the existing models will use the traditional multi-scale filtered convolutional neural network (CNN) to obtain simple word vector features in the process of text classification. Although this model attaches importance to word vector, it ignores other important features of semantics itself. On this basis, they proposed a short text classification model based on CNN, The nonlinear sliding method and *n*-gram language model are used to obtain rich text features, and the centralized mechanism is used to extract key features and retain the most determined text features [7]. Ma et al. discussed bilingual rotation in the context of neural machine translation proposed an interpretation model based on a neural network, and generated candidate interpretation for Arabic etymological input. The results showed that neural interpretation was significantly better than statistical machine translation, and there was a high similarity and correlation between the model and human translation [8]. Petrucci et al. proposed a coding and decoding system based on neural network, which converts natural language definitions into descriptive logic formulas through syntactic conversion, so as to evaluate its generalization ability in different syntactic structures, tolerate unknown words, and improve its performance by enriching the training set with new annotation examples [9]. Farzi et al. introduced a neural reordering model in their research, using a phrase dependency tree that describes the dependency relationship between continuous nonsyntactic phrases, using reordering rules and performing long-distance reordering, combining the functions of lexical reordering and syntactic presorting models [10]. Sentence regression is a type of abstract extraction, which can achieve the most advanced performance, and is usually used in practical systems. In the sentence regression framework, the most challenging task is to identify the distinctive features representing each sentence. Ren et al. proposed a deep neural network model - sentence relation-based summary (srsum) in their research on the use of sentence relations. When studying the semantic analysis of natural language translation, priorsum uses double graph convolution neural network to encode the potential semantics of sentences, sfsum encodes the surface information of sentences, and csrsum tsrsum and QSR sum are three sentence relation sub models [11].

To sum up, it can be seen that there are many pieces of research on translation neural networks, most of which adopt the general model based on neural network. Although this standard forward feedback neural network is relatively mature, the prediction model defaults that there is a certain connection between the translated documents to a certain extent, has a strong dependence on structural analysis, ignores the value of semantics itself, and the English character image itself is more complex. In the training process, although the local optimization method can be adopted, it needs multiple calculations, and the calculation of each step will affect the subsequent analysis. Therefore, there will be the problem of wrong translation, and if there is poor convergence, it is easy to fall into the local optimal solution. Although neural network is widely used, its standard structure is not suitable for all English translation. Therefore, it is of great practical significance to carry out the research on semantic analysis technology of English translation based on deep neural network.

## 3. Methodology

### 3.1. Translator Framework

In the language-translation encoder, different from other deep neural networks, the mainstream mode belongs to the sequence-to-sequence mode. This model appears earlier. The background information is input into the decoder. After passing through the encoder, all the information becomes the target language sequence [12]. The specific framework is shown in Figure 1.

The framework is a classical neural network translator model framework, which is relatively mature. The output sequence of the encoder is called context, and the vector is represented by *C*. the input vector is the output vector of the encoder and also the input vector for the decoder [13]. The decoder outputs in the form of probability, which is predicted according to the previous output. The formula is as follows:

(1) $$\begin{array}{c} p\left(y\right)=\prod_{t=1}^{T_{y}}P\left(y_{t}|y_{1},y_{2},\ldots ,y_{t-1},C\right),\\ p\left(y_{t}|y_{1},y_{2},\ldots ,y_{t-1},C\right)=g\left(y_{t-1},h_{t},C\right), \end{array}$$

where *T* represents the length of the output sequence. This encoder-decoder structure is the framework commonly used in neural machine translation. In this paper, semantic translation is also based on this framework.

### 3.2. Neural Network-Based Depth Translator

Most common translation machines are based on linguistic knowledge. The translator based on a deep neural network focuses on the design of neural network structure [14]. In practical application, different neural networks will directly affect the translation effect. Among various network structures, cyclic neural networks are widely used, which can store timing information and process input sequences of any length [15]. The information output from each layer of the cyclic network reaches the next layer, which is represented by the state parameter function of the hidden layer, which can effectively deal with the dependent translation information [16]. In the single hidden layer feedforward neural network, the hidden layer activation function is expressed by the vectorization method. Assuming that the hidden layer length is *h* and the feature vector dimension is *x*, the hidden layer output formula can be expressed as:

(2) $$\begin{array}{c} H=\delta \left(XW_{xh}+b_{h}\right),\\ \text{sigmoid}\left(x\right)=\frac{1}{1+e^{-x}}, \end{array}$$

where *X* represents the batch data, *W*_*xh*_ represents the input weight parameter of the hidden layer, and *b*_*h*_ represents the offset vector parameter. The parameters of the weight vector and offset vector are calculated by broadcast data. Assuming that the output vector dimension corresponding to the sample is represented by *Y*, the final output can be expressed as:

(3) $$\begin{array}{c} \overset{\wedge }{Y}=\text{softmax}\left({\text{HW}}_{ky}+b_{y}\right),\\ \text{softmax}\left(x_{m}\right)=\frac{e^{x_{m}}}{\sum_{k}e^{x_{k}}}. \end{array}$$

The encoder converts the source language sequence into word vector data, transmits it to the neural network, saves it to the background vector, and finally inputs the target language sequence [17]. When it is transformed into a cyclic neural network, the time stamp needs to be added. When calculating the hidden layer, the hidden layer state output can be obtained according to the vector. The formula is expressed as:

(4) $$\begin{array}{c} H_{t}=\delta \left(X_{t}W_{xh}+H_{t-1}W_{hh}+b_{h}\right), \end{array}$$

where *W*_*xh*_ represents the newly introduced weight parameter, and the output result can be obtained according to the formula. The formula is as follows:

(5) $$\begin{array}{c} \overset{\wedge }{Y}=\text{softmax}\left({\text{HW}}_{hy}+b_{y}\right). \end{array}$$

In the cyclic neural network, all the output values of the network are the network information values in this state. In the application, this information needs to be expressed in the form of word vectors, and then these word vectors are used as the input information [18]. In the whole training process, if the time series training sample size is large or small, the hidden layer may have gradient attenuation. In the calculation of deep neural network, the back-propagation method needs to calculate the chain derivative, and each calculation needs to be multiplied. If the silver is less than 1, the result will not tend to 0, gradient attenuation will occur, and the subsequent parameters cannot be updated [19]. However, if it is greater than 1, the result will be large and prone to gradient explosion. It is necessary to cut the gradient, splice a vector, and limit the size of the threshold through the following formula:

(6) $$\begin{array}{c} g=\min\left(\frac{\theta }{\left|g\right|},1\right)g, \end{array}$$

where *θ* represents the threshold and *g* represents the vector of gradient splicing. It should be pointed out that although time gradient clipping can solve the possibility of gradient explosion, gradient attenuation will still occur. Therefore, this algorithm cannot deal with the problem of long-distance dependence, and other algorithms need to be adopted [20]. The neural network structure based on long-term and short-term memory needs to determine which information to forget first. To overcome the weakness of traditional RNN, short-term and long-term memory network (LSTM) combines short-term memory and long-term memory through gating and effectively solves the problems of gradient disappearance and gradient explosion in RNN prediction network. Through deep learning and long-term memory ability of information, control the degree of information attenuation. Suppose that at a certain time, the number of samples is *n*, the hidden layer state at the previous time is represented by *H*_*t*−1_, and the forgetting gate can be expressed as:

(7) $$\begin{array}{c} f_{t}=\delta \left(X_{t}W_{xf}+H_{t-1}W_{hf}+b_{f}\right), \end{array}$$

where *W*_*xf*_ represents the learning weight parameter, *b* represents the paranoid vector parameter, and the broadcast data operation is used to calculate the vector. Then select the information to be retained, update the value, and then use the hyperbolic tangent function to generate the candidate set. The formula is expressed as:

(8) $$\begin{array}{c} i_{t}=\delta \left(X_{t}W_{xi}+H_{t-1}W_{hi}+b_{i}\right),\\ \overset{-}{C_{t}}=\tanh\left(X_{t}W_{xc}+H_{t-1}W_{hc}+b_{c}\right). \end{array}$$

This step is the same as the previous step to calculate the weight parameters. Then update the memory unit status. In this process, use the old status multiplied by the forgotten information to update. This step combines the current memory unit information and the memory unit in the previous step. The formula can be expressed as:

(9) $$\begin{array}{c} C_{t}=f_{t}⊗C_{t-1}+i_{t}⊗\overset{-}{C_{t}}. \end{array}$$

It can be seen from the above formula that if the input gate is approximately 0 and the forgetting gate is approximately 1 at the same time, this memory unit will always be maintained, so there will be no gradient attenuation, and the dependency in the time series can be well analyzed [21]. After the memory unit is updated, the output controls the flow of the memory unit, and the sigmoid layer determines the output memory unit. The formula is as follows:

(10) $$\begin{array}{c} o_{t}=\delta \left(X_{t}W_{x0}+H_{t-1}W_{h0}+b_{0}\right),\\ H_{t}=o_{t}⊗\;\tanh\left(C_{t}\right). \end{array}$$

When the output gate is 1, the information is transferred to the hidden layer. If it is 0, the memory unit information will be saved.

In the process of English translation, the translation of words cannot be taken literally, and the meaning of context needs to be comprehensively considered. Compared with other learning algorithms, the training neural network can scan information for storage and process context information. Although it has great advantages, it also has its own disadvantages and will not consider the change of specific information [22]. Therefore, the bidirectional cyclic neural network is used in this analysis. This algorithm uses cycles in different directions to scan the information sequence, generate different hidden layer sequences, and then splice them. In this structural design, the neural network passing in two directions can be passed forward or backward. The forward neural network scans from front to back to generate the forward hidden layer sequence [23]. When scanning backward Gru neural network, the input sequence is scanned from back to front to generate the reverse hidden layer sequence. The two hidden layer sequences are spliced to form the language terminus $h={\left[{\overset{⟶}{h}}_{i}^{T},{\overset{\leftarrow }{h}}_{i}^{T}\right]}^{T}$. Through this design method, the context information can be included without losing part of the sequence information.

### 3.3. Translation of Part of Speech Sequence Information

At present, the common translation neural machines generally adopt end-to-end methods to realize the mapping between the target language and the translation language, which can play a certain effect in simple machine translation. However, some neural network structures are not nonlinear and it is difficult to use a priori knowledge for translation. Therefore, this translation model needs to be further improved, so the part of speech sequence information. The neural machine maps the translation language into input sequence information, and then generates the target language [24]. In this process, all the information and features of the translated language will be saved in the background vector. Background vector can transfer semantic information, so integrating more language knowledge into the background vector can effectively improve coding efficiency and translation effect. While encoding, store the information as a priori knowledge into the background vector to jointly realize translation training [25].

When analyzing the part of speech sequence information, we need to analyze the information of language sentences, judge the composition of the input word sequence, analyze the structure and the relationship between word components through the structure, and determine the composition, function, and grammatical problems of words. After coarse-grained processing of language structure, a part of the speech sequence classification model consisting of four notional words, noun verbs, adjectives, and pronouns, is constructed. The results show that the accuracy of the natural language part of the speech sequence classification model based on part of speech content reaches 90%. The classification model of the natural language part of speech sequence based on word order position has high accuracy. The part of the speech sequence classification model of natural language has good application value in the field of language cognition. It can not only reveal and confirm the relationship between language and psychological information but also scientifically evaluate the implicit psychological information through objective language symbols. In the analysis of sentence sequence information, there are mainly two forms: prestored syntax and phrase structure, in which the prestored syntax directly reflects the relationship between sentences and words. At present, there are many syntactic analysis tools commonly used. Stanford parser is a kind of commonly used tool, which can analyze words that are not related to context and Related words. This tool is used in syntactic analysis. By inputting the syntactic information into the translation model, the relationship between words in the sentence can enter the background vector at the same time. Under this operation, the dependence on distance can be reduced. If the part of the speech sequence is continuous, we can also get the desired results of sentence structure analysis.

Based on bidirectional Gru neural machine translation, the part of speech sequence information is integrated to construct the part of speech model of neural and its translation, as shown in Figure 2. The source language input information in the figure is encoded, and the encoded information at any time is combined by vector splicing. Input the text that needs to be translated into it. After the step of word embedding, the word embedding can convert the language information into numerical form, then encode the input word and encode the position information. Input this information into the encoder, and the encoder transmits the information to the decoder. The input step of the decoder is the same. For the source language input sequence, the hidden layer can be obtained. Similarly, for the part of speech sequence information, the hidden layer state sequence can also be obtained. For different sequences, concat is carried out for each word to calculate the background vector.

## 4. Result Analysis and Discussion

### 4.1. Model Simulation Analysis Based on Bidirectional GPU Neural Network

This paper studies the application of semantic analysis based on deep neural network in English translation. The transformer is introduced from the perspective of industrial practice. Wmt2018 global machine translation evaluation results are used for analysis and research. Before using neural network for English translation, we need to preprocess the data and analyze the feasibility of neural network model machine translation. To measure the network performance, the neural network is used for simulation analysis to measure the complexity and running time. In the training, the randn function is used to control the noise information, and the change of error rate of the common neural network and RNN neural network is analyzed. The comparison and analysis results of the recognition error rate are shown in Figure 3. From the data changes in the figure, it can be seen that after adding noise data, the translation error rate of the two neural network models has improved, but in comparison, the deep neural network model proposed in this paper has better performance in resisting noise data.

When analyzing the translation performance of deep learning network model, it is generally believed that the larger the data scale, the better. Combined with the actual situation, in the simulation analysis, iwslt database is selected. This database has a smaller scale, but it is also a database commonly used in international translation, which can also be used to measure translation performance. The bidirectional Gru neural network model algorithm proposed in this paper is compared with the traditional model algorithm (such as RNN model, Gru model, and LSTM model). The development set data and test set data are 1 pair and 3 pairs respectively, the word vector dimension is 512, the number of hidden layer nodes is 512, and the learning rate is set as 0.1. The baseline translation model adopts the niutrans model based on shorter than, and bleu-4 value is used in the evaluation of translation effect.

Different neural networks are used to test the training set respectively. The translation results are shown in Figure 4. From the data in the figure, it can be seen that the translation score of niutrans is the highest in the development machine and training set, which is a relatively mature translation model. In contrast, GRU structure also has certain advantages and its performance has been improved, which shows that the bidirectional GRU neural network model proposed in this paper has certain advantages in English translation. The performance of the two is equal in many tasks. It is easier to converge with fewer Gru parameters, but the LSTM performance is better when the data set is large. Gru has only two gates (update and reset), and LSTM has three gates.

In the analysis of the performance index of the translation model, the confusion degree is used for evaluation. This index reflects the reciprocal of the average probability of word semantic translation. Train the global word vector on the training set and calculate the degree of confusion. The hidden layer size is set to 100 and the window length is 50. The comparative analysis of chaos is shown in Figure 5. From the data changes in the figure, we can see that the translation performance increases with the increase in vocabulary. With the increase of dimension, the performance becomes better, indicating that the translation can obtain information in combination with the context.

Neural network model can solve the problem of data coefficients, but it also has its disadvantages in long-distance information description. Therefore, in this paper, different neural network models are applied to word vector analysis, and the feature layer adds a context transfer vector to improve the learning ability of information constraints. Analyze the changes of translation performance under different hidden layers, set the word vector dimension to 50. The effect of the hidden layer on confusion is shown in Figure 6. It can be seen from the figure that after the introduction of word vector, the translation performance of deep neural network model has been improved. In contrast, when the number of neurons increases, the performance superiority of the bidirectional GRN model is more obvious.

### 4.2. Model Simulation Analysis of Adding Part of Speech Sequence Information

This paper compares and analyzes the translation effects of translators after adding part of speech sequence information. Taking transformer model as the research object, syntactic information is integrated into machine translation model. The source code of transformer model is deeply analyzed. On this basis, the dependency information at the source end is obtained by establishing a dependency tree for the source language sentences. According to the dependency information guidance of the source side, we can obtain more abundant relevant information between words and sentences on the source side. The word with the greatest relevance to the current word is selected as the word of attention distribution. In this way, we can integrate syntactic dependency information. The improved system has better translation performance and can further improve the quality of translation. It is compared with the baseline translator. In the setting of magic training parameters, the architecture is the same and the parameter settings are the same. Except for adding part of speech sequence information, other information is the same. In the data set selection, using the English corpus, select two vocabulary sets with different sizes, and the total sample contains thousands of word sentence pairs.

The Open-Source Toolkit Spacy and the original sequence are used to extract part of speech tagging and store it in the data set. The batch size is set to 128. The encoding and decoding are three-layer structure, the hidden layer size is 256, and the complete training sample is 10. The translation performance and error values of the part of speech sequence information model, LSTM model, RNN model, and two-way RNN model are measured. The comparative analysis of translation performance is shown in Figure 7. From the data in the figure, it can be seen that the improved translation algorithm can improve the Bleu value, the error value does not change significantly in several models, the experimental effect is better, and the translation effect is improved.

The change of loss function reflects the convergence of the algorithm, so it is necessary to measure the change of loss function under different models. In the measurement, the changes in loss function of part of speech sequence information model, train model, and rnnlm model are analyzed under different iteration times. The change of loss function is shown in Figure 8. From the data change in the figure, it can be seen that the loss function in rnnlm model decreases relatively slowly. After adding part of speech sequence information, the convergence speed of loss function decreases faster, but the convergence effect is better than that of the traditional algorithm. Because of the part of speech sequence information, the dependence on the number of training samples is greatly reduced, and the training efficiency is improved.

In English sentence analysis, in addition to analyzing semantic information, we also need to pay attention to word segmentation and syntactic composition, otherwise, the translation efficiency will be greatly reduced. In the test of the model based on deep learning network, the translator is used for translation, the random gradient descent method is used to optimize the parameters, and the translation performance results are compared and analyzed. Compared with the baseline system, after adding semantic information, the Bleu value of the translation model increased from 23.5 to 23.7, indicating that this method can improve the translation performance.

The translation machine based on neural network is sensitive to length, and its performance will reach the best value only after reaching a certain length. To make full use of the massive parallel corpus, this paper considers the sentence length information of the parallel corpus and divides the original parallel corpus into several modules. A submodel is trained for each module, and a neural machine translation method based on sentence length fusion strategy is proposed. When the training is finished, the translation is obtained by the model fusion after sentence length boundary division and the three features (confusion degree, sentence length ratio, and classifier) fusion sorting method. To analyze the translation effect after adding semantic information, sentences with different lengths are classified and translated. The sentence length is divided into five categories. The translation performance differences of part of speech sequence information model, niutrans model, and bigrnn model are measured. The measurement results are shown in Figure 9. It can be seen from the data changes in the figure that the translation performance is improved after the sentence length increases, and no matter what the length of the sentence, the performance of the translation model with semantic information is the best, and this advantage becomes more obvious with the increase of the sentence.

## 5. Conclusion

With the increasingly frequent exchanges between different countries and industries, machine translation has received extensive attention. Machine translation can realize language translation based on retaining the original semantics. The application of a neural network also greatly improves the translation performance, greatly simplifies the translation process, and improves the efficiency, but it is still unable to contact the context, and the semantic translation is wrong. Based on this, this paper studies the application of semantic analysis of English translation based on deep neural network. Aiming at the shortcomings of neural network translation, this paper designs a neural network model framework, makes full use of word vector in the construction of language sequence, and puts forward a neural machine translation model of two-way Gru for the shortcomings of the traditional neural network model, and introduces word sequence information, The performance of the translation model is verified by the in-depth simulation of the neural network.

However, the study still has some limitations. The scale of data used in research and analysis is reduced, and it is difficult for training data to use large-scale data for simulation analysis, which may affect the performance analysis results of deep learning network model. Therefore, further modifications are needed in the future research. In improving English semantic analysis, we can consider further improvement from the perspective of model memory ability, interpretability of translation, constraint ability of prior knowledge, and so on.

## Figures and Tables

**Figure 1:** Specific frame diagram.

**Figure 2:** Transformer model design with part-of-speech information vector added.

**Figure 3:** Comparative analysis of recognition error rate.

**Figure 4:** Comparative analysis of translation model performance.

**Figure 5:** Comparative analysis of confusion.

**Figure 6:** Influence of hidden layer on confusion.

**Figure 7:** Comparative analysis of translation performance.

**Figure 8:** Variation of loss function.

**Figure 9:** Comparison of translation of sentences with different lengths.

## Data Availability

The data used to support the findings of this study are available from the author upon request.
